The article "Assessing the impact of water scarcity on thermoelectric and hydroelectric potential and electricity price under climate change: Implications for future energy management" was published in 2024. Journal: Heliyon.

# Assessing the impact of water scarcity on thermoelectric and hydroelectric potential and electricity price under climate change: Implications for future energy management

**DOI:** 10.1016/j.heliyon.2024.e36870

**Published:** 2024-08-29

**Authors:** Qiang Guo, Reza Hasani

**Affiliations:** a School of Management, Xinxiang University, Xinxiang, 453003, Henan, China; b Islamic Azad University Central Tehran Branch, Tehran, Iran; c College of Technical Engineering, The Islamic University, Najaf, Iraq

**Keywords:** Water resource limitations, Hydroelectric, Thermoelectric, General circulation models, Echo state network, Modified snow leopard optimization algorithm

## Abstract

This study investigates the impact of water resource restrictions on thermoelectric and hydroelectric stations, analyzing its influence on demand and electricity prices. It uses General Circulation Models (GCMs) and Soil and Water Assessment Tools (SWAT) to forecast future temperature trends and estimate river flow patterns. The research provides insights into climate change's potential effects on water resources and electricity potential. The study shows a significant decrease in river flow, indicating potential issues with hydroelectric and thermoelectric systems. The study also uses an optimized Echo State Network (ESN) for accurate electricity demand, using the Modified Snow Leopard Optimization (MSLO) algorithm as a new metaheuristic model. The simulation results show a consistent increase in electricity demand scenarios, which is expected to lead to higher supply prices due to decreased production capacity. This could have significant economic effects. The investigation provides a comprehensive understanding of water resource management challenges in power production, aiding in informed decisions in the future energy industry.

**Table:** 

**Abbreviation**		**Nomenclature**	
SWAT	Soil and Assessment and Tools	$SW_{T}$	the final soil water content
RCPs	Representative concentration pathways	$SW_{0}$	the initial soil water content
MSLO	Modified Snow Leopard Optimization	$R_{i}$	precipitation
ENS	Echo State Network	$Q_{surf,i}$	surface runoff
GCM	The General Circulation Model	$E_{i}$	evapotranspiration
CMIP6	Coupled Model Intercomparison Project Phase 6	$Q_{lat,i}$	lateral flow
IPCC	The Intergovernmental Panel on Climate Change	$Q_{rev,i}$	return flow from irrigation
GHG	Green-House Gas	$P_{h}$	the available power
DCSA	Developed Crow Search Algorithm	ρ	Water density
IECM	Integrated Environmental Control Model	q	the water flow rate
CanESM5	Canadian earth system model version 5	g	the acceleration due to gravity
SSPs	Shared Socioeconomic Pathways	h	head
TEGs	Thermo-Electric Generators	μ	efficiency of the hydropower system
SLO	Snow Leopard Optimization	$P_{a}$	the hydropower available
GSA	Gravitational Search Algorithm	$P_{T}$	thermoelectric power output
SSA	Squirrel search algorithm	μ	the water availability factor
BBO	Biogeography-Based Optimizer	η	the thermoelectric efficiency
MSE	The Mean Squared Error	S	the Seebeck coefficient
SD	Standard deviation	V/K	volts per kelvin
MVO	Multi-Verse Optimizer	σ	electrical conductivity
MAPE	Mean Percent Fundamental Error	κ	thermal conductivity
Avg	Average	T	the average temperature
RMSE	Root Mean Square Error	AF	activation function
MAE	Mean Absolute Error	P	the expected output
DEM	Digital Elevation Model	$\hat{P}$	the actual output
ESP	the Echo State Property	$T_{h}$	the hot side temperature
SR	Spectral Radius	$ZT_{h}$	dimensionless

## 1 Introduction

### 1.1 Background

Hydroelectric and thermoelectric power plants have significantly contributed to China's electricity production and make water-energy security an increasingly crucial challenge not just in China but also worldwide [1]. Water and electricity generation are closely linked, and these two topics are interlaced. Power plants that use thermoelectric generation withdraw water from rivers or lakes to cool their units and then return warmer water to the original water source. Hydropower is the direct utilization of water flow to produce renewable power, which is fueled by solar energy that drives the hydrologic cycle. The electricity sector relies heavily on the accessibility and temperature of water resources for both hydropower generation and cooling of thermoelectric power plants [2]. The availability of water resources on Earth is crucial in determining the potential for generating hydropower and thermoelectric power [3]. As the global population continues to grow and economies develop, electricity demand is expected to rise, which will be affected by changes in surface water resources.

Due to the impact of global warming and climate change, the significance of water resource management has grown significantly in recent times. This is because of the increase in severe climatic changes such as floods and storms. Environmental concerns have become a top priority and prompt the development of sustainable solutions. It is essential that the availability of hydropower in many areas is reliant on weather patterns, and changes in climate will impact the hydropower resource and its generation. It is possible that in several areas across the globe, the change in climate will lead to a reduction in water supply while also causing a detrimental impact on water quality and temperature [4]. The changes in water resources caused by climate change will have a direct impact on the link between water and energy [5] and result in a decrease in the production of electricity. As a result, all water users, water providers, and water management systems will be affected.

Climate change has a significant impact on the energy sector due to its direct influence on water quality and quantity, which is a critical factor in electricity generation [6]. Due to its reliance on water for electricity generation, the energy sector is highly susceptible to variations in water quality and quantity caused by climate change. Water scarcity or rising river temperatures due to climate change are affecting thermoelectric power industries in many countries today. Thermoelectric power plants typically extract the water required for cooling from either rivers or the ocean [3]. The use of water for cooling power plants may be endangered if the rivers’ temperatures become too high or the stream flow is too low. This is not because of physical laws but due to the possible violation of water quality regulations [7]. So, the efficiency of the cooling process can be reduced due to high temperatures [8].

Water is an essential resource for cooling in coal-fired and nuclear power plants. The thermoelectric energy sector, which mainly involves generating electricity from thermal power plants, consumes more water than any other sector, including industry, agriculture, and domestic usage. Surface water resources are significantly withdrawn by this industry. Thermal power plants require water resources for various stages of electricity production, such as cooling, steam generation, and flue gas desulfurization. Approximately 60 % of the water consumption in the power industry is attributed to the production of Coal-based energy [9]. Ensuring sustainable utilization of the valuable resource of water is of utmost importance, particularly in the power sector, where its consumption is a significant concern and needs immediate attention.

The consumption of electricity is affected by climate change as the fluctuating temperature alters the heating and cooling requirements of individuals [10]. During winter, countries with colder climates tend to decrease their energy consumption for heating as the temperature increases. The availability of water in China has been negatively impacted by global warming, climate change, and rising temperatures, which has elevated the risk of the production of electricity. A significant decrease in hydroelectricity generation has led to a severe water supply shortage for the thermoelectric cooling system, which is negatively impacting the general energy supply of the country.

The demand for energy in economies is rising due to economic growth and population increase. The energy demand of an economy is influenced by the economic growth rate and the energy efficiency of the production sectors [11]. Technological advances impact the energy intensity of different industrial sectors. The demand for electricity is on the rise due to the fast-growing world population, which in turn leads to an increase in electricity prices. It is crucial to analyze the impact of limited water resources on the generation of thermoelectric and hydroelectric power and understand how it affects the demand and cost of electricity. An increase in the price of electricity supply is expected due to the rising demand for electricity, which is a key discovery of this study. The economic impact of the widening gap between electricity supply and demand could be significant. As a result, it is crucial to adopt a holistic approach to energy production and distribution that meets the increasing demand while also being both cost-efficient and sustainable. There have been various studies regarding this topic, some of which will be discussed in the following section.

### 1.2 Literature review

Zhang et al. [12] conducted a study whose purpose was to illustrate the current situation and further changes in thermoelectric usage and stress of water in India. The geographical database of entire thermal plants that, was a bottom-up technique were collected. Moreover, the technology kind for cooling was recognized. The thermoelectric extraction of and consumption of water were anticipated between the years 2009 and 2018. Then, further changes within thermoelectric usage of water were anticipated by 2027 by the use of combined planning of power and model dispatch. The outcomes indicated that thermoelectric production of power was not considered to be the main stress source of water by 2027 in India. In addition, the extraction of fresh water was different in the range of 14 and 16 billion $m^{3}$ within the period of investigation, whereas the usage of freshwater rose to the growth thermal production of water. The catchment existing within the Ganga River possessed the greatest extraction of fresh water and usage. The amount of extraction of water was less than 1 % of freshwater accessibility that existed in catchments. In the upcoming years, a major amount of extraction of water and power production would probably happen within the catchments whose stress of water is inferior. Focusing on areas with high water stress, it is important to implement rule interferences that enhance the stability of thermal power manufacturers against outages caused by the stress of water.

Voisin et al. [13] implemented research and assessed the way that estimated alteration of the water accessibility influenced the production of energy from thermal and hydroelectric power plants. Moreover, it was investigated how the corresponding effects propagated the neighborhood and all through the energy grid that was interlinked in the western United States. The fact that the climate alteration had the capability to influence the energy reliance of the region was assessed. The imitations of hydrology derived from radiative circumstances (RCP8.5 and RCP4.5), a model of the VIC hydrology, and three international distribution models (INMCM4, GFDL-CM3, and CCSM4) were utilized for driving a circulated and large-scope management model of water (MOSART-WM) rendering accessibility of water into restrictions of energy production at thermoelectric plants of water-reliance and hydropower plants. The dynamics of the energy system were assessed by the utility of the expense model of generation, PLEXOS. It was found that inter-territorial links in the current energy substructure of the country had a pivotal role in management differences in local production because of hydrological inconsistency. The alterations in the average annual precipitation across the WECC region, with a range between −3.8 % and +17 %, were mitigated to a range between −6% and +4 % when it came to the changes in the average annual generation expense. Effects of change in climate on the accessibility of water in the Northwest caused further trends within a generation of other areas and in local flows of power. The entire production of Northwest impacted inter-annual inconsistency in net production of other areas that depicts variability of approximately 50 %, 35 %, and 40 % in Rockies, Southern, and Southwest California regions, respectively. The climate alteration influence of Northwest on the grid was intensified through the incidence of years that were dry in Northern California. Production of Southwest Desert appeared to be an important resource in order to make up for differences in production and accessibility of water within the current areas.

Terrapon-Pfaff et al. [14] carried out an investigation that illustrated suggestions of undetermined techniques of decarburization for the direct demand of water for energy production. In doing so, situations of water demand for energy segmentation were created on the basis of international electricity research for analyzing the effect systematically by 2040. The findings illustrated that various techniques of decarburization for energy segmentation might result in an extensive disparity in the requirements of water. Decreasing emissions of Green-House Gas (GHG) did not result in a decline in the demand for water. The outcomes highlighted the necessity for considering the emission decrease of greenhouse gas and various facets like the demands of water for upcoming electricity systems. The consideration was conducted at global and local degrees for accomplishing a renewable energy alteration.

Huangpeng et al. [15] suggested a method with the aim of forecasting the future generation of hydropower (2021–2050) regarding climatic changes. The Developed Crow Search Algorithm (DCSA), in combination with ANN models, was utilized to enhance the precision of flow estimation in this investigation. The approach implemented in this study included the adoption of the latest version of DCSA (Developed Crow Search Algorithm). The optimization weaknesses, including being stuck in the optimum position and the imbalance between exploration and exploitation at various levels, could be resolved by this algorithm that, resulted in increased prediction accuracy. According to the findings, the DCSA algorithm exhibited the best performance compared to other algorithms, with the least error (MSE = 1.06) and the highest correlation (R^2^ = 0.88). The forecast results for climate change scenarios using RCPs indicated that the average annual **power** generation would experience a decrease of approximately 10.74 %, 16.38 %, and 22.25 % under RCP2.6, RCP4.5, and RCP8.5, respectively. Additionally, by 2050, the average annual power generation under RCP2.6, RCP4.5, and RCP8.5 scenarios were forecasted to be 740.33 MW, 603.12 MW, and 585.77 MW, respectively.

The objective of Shinde et al. [16] was to measure how much climate change affected the within-year water stress that thermal power plants in India face. In order to measure monthly water withdrawal and consumption for thermal power plants in four water-stressed states of India, the Integrated Environmental Control Model (IECM v11.5) was utilized. The range of water withdrawal was between 2400 and 5500 L per megawatt hour, and it experienced an increase of up to 24 % during the summer season in comparison to the winter season. Two climate change scenarios, SSP2 – RCP 4.5 and SSP5 – RCP 8.5, were simulated and indicated a rise of 7–18 % in water withdrawals as compared to the existing levels. Future surface water availability in Rajasthan was expected to decrease by over 49 % for both scenarios as compared to estimated using Budyko's framework. Careful planning would be necessary to manage climate change impacts in the future since power plants in the regions analyzed would face water deficits during January–May.

### 1.3 Motivation

An examination of the literature review has identified a significant gap in the used models, including climate models and neural networks, in accurately forecasting the impacts of limited water resources on electricity generation and consumption. Given these limitations, there is a requirement for a more sophisticated framework to address these issues and offer a thorough analysis of the effects of water scarcity on supply and demand. By emphasizing the necessity of a detailed exploration of the potential impact of climate change on water resources and electricity production, this study seeks to bridge this divide and provide valuable insights in this area. The emphasis on understanding the repercussions of global warming on water availability and its subsequent influence on hydropower and thermoelectric generation highlights the significance of this research in tackling crucial research gaps in the field.

### 1.4 Contribution

This investigation aims to evaluate how hydroelectric and thermoelectric potential might be affected by water resource limitations and how this could impact electricity demand and electricity price. The study utilizes advanced modeling techniques, including the General Circulation Models (GCMs) and the Soil and Water Assessment Tools (SWAT) hydrological model, to gain insights into the expected impact of global warming on water resources. The research findings are expected to provide valuable insights into the implications of water resource limitations resulting from global warming on electricity potential. Accurate demand forecasting is a crucial element in the management of resources and the determination of electricity prices effectively. To achieve this, the study utilizes an optimized forecasting approach that combines the Echo State Network (ESN) with the innovative Modified Snow Leopard Optimization (MSLO) algorithm. This method enables energy analysts and policymakers to plan future electricity consumption more precisely by providing more accurate predictions of electricity demand trends. Developing sustainable energy strategies and ensuring a reliable and affordable electricity supply can be facilitated by using the insights provided by this research, which can guide the decision-making processes in the energy sector.

• The impact of water resource constraints on thermoelectric and hydroelectric potential.
• To forecast future temperature trends employed General Circulation Models (GCMs).
• Soil and Water Assessment Tools (SWAT) estimates the flow patterns.
• Optimized Echo State Network (ESN) has resulted in accurate electricity demand.
• The Modified Snow Leopard Optimization (MSLO) algorithm optimes ESN model.

The paper initiates with Section 1, the Introduction, offering an outline of the study's background, objectives, and contributions. Following this, Section 2, Method and Material, elaborates on the research methodology, which includes case studies, data descriptions, and various simulations related to temperature forecasting, river flow predictions, and electricity demand and pricing models. Progressing to Section 3, Results, the document showcases the results of the research conducted, covering findings on temperature forecasts, hydropower potential, and the effects of climate changes on electricity demand and prices. Lastly, in Section 4, Conclusion, the key insights and implications of the study are summarized, providing a cohesive conclusion to the document.

## 2 Method and material

### 2.1 Case study and data description

Yunnan, located in the southwestern region of China, boasts a varied landscape and climate. The average annual temperature ranges from 8 to 23 °C, varying based on altitude and latitude. The monsoon circulation greatly influences Yunnan, resulting in a dry season from November to April and a rainy season from May to October. With a subtropical monsoon climate, the province receives an annual rainfall ranging from 560 to 2300 mm, mostly occurring between June and August [17].

The information required to forecast the demand and price of electricity is sourced from two distinct platforms. Firstly [18], provides the latest international trade data for Yunnan Province, including the exports and imports of various products and destinations. Secondly, the gross domestic product (GDP) of Yunnan Province from 2012 to 2022 and other economic indicators and statistics have been collected from Ref. [19]. Additionally, the prices and values of Yunnan coins graded by two professional coin grading services, PCGS and NGC, have been obtained from Refs. [20,21].

The province is rich in hydropower resources, possessing a reserve of 202.4 million kW and a technically exploitable capacity of 103.6 million kW. Additionally, Yunnan exhibits immense potential for thermoelectric generation. A study suggests that by 2030, Yunnan's thermoelectric power generation could reach 1.8 GW. Yunnan experiences four distinct seasons, characterized by mild winters and warm summers. Yunnan supplied 75.8 billion kWh of electricity to other provinces [22].

The Xiangjiaba hydropower plant has been examined in this research to predict its power potenrial in the face of climate changes. This project, which is situated on the Jinsha River, a tributary of the Yangtze, in China, has a capacity of 6.4 GW. It is equipped with eight 800 MW Francis turbines and three 450 MW turbines, resulting in a total installed capacity of 7.75 GW. The plant generates an average annual power output of 30.747 TWh [22].

Fig. (1) show the Yunnan province location.

**Fig. 1:** The Yunnan province location in China.

The methodology flowchart has been shown in Fig. (2).

**Fig. 2:** The methodology steps.

### 2.2 Temperature forecasting by Global Climate Models (GCMs)

Global Climate Models (GCMs) are advanced instruments that replicate the interactions between different elements of the Earth system, such as the atmosphere, ocean, land, and sea ice. They have a vital function in forecasting future fluctuations in worldwide and local mean surface temperatures by taking into account various scenarios associated with socioeconomic progress and greenhouse gas emissions. CanESM5, a well-recognized model, is extensively used for temperature prediction, specifically within the framework of the 6th phase of the Coupled Model Intercomparison Project (CMIP6). The Canadian earth system model version 5(CanESM5) model is a comprehensive computational tool that actively engaged in the CMIP6 simulation, facilitating the execution of coordinated climate experiments across many Representative Concentration Pathways (RCPs) and Shared Socioeconomic Pathways (SSPs). The RCP-SSP scenarios combine Representative Concentration Pathways (RCPs) and Shared Socioeconomic Pathways (SSPs) to describe the potential evolution of climate forcing and human society in the 21st century. The SSP-RCP scenarios represent different radiative forcing levels and socioeconomic development, such as RCP2.6-SSP1, RCP4.5-SSP2, RCP8.5-SSP5, etc. The paths RCP2.6, RCP4.5, RCP8.5, SSP1-2.6, SSP2-4.5, and SSP5-8.5 include a range of radiative forcing values spanning from 2.6 to 8.5 W/m^2^ by the conclusion of the 21st century.

Additionally, these entities embody distinct socioeconomic development paths, including sustainability, moderate progress, regional competition, inequality, and development reliant on fossil fuels. By examining these scenarios, General Circulation Models (GCMs) such as CanESM5 provide significant contributions to the understanding of climate patterns and aid in forecasting forthcoming alterations in worldwide and local temperatures. These predictions are derived from a range of assumptions pertaining to socioeconomic variables and greenhouse gas emissions.

In this study the GCM model (CanESM5) forecasts the climate parameter (temperature) under RCP-SSP scenarios. The temperature is used as one of the effective input parameters in the SWAT model to forecast future changes in river discharge.

### 2.3 The flow river forecasting under climate changes

Predicting future changes in river discharge under climate parameter changes (temperature) using the SWAT model involves projecting the river's flow based on different assumptions about socioeconomic development and greenhouse gas emissions.

The SWAT is a hydrological model that can simulate various aspects of water balance in a watershed, such as surface runoff, groundwater flow, and water quality. To make these simulations, it utilizes meteorological, soil, land use, and topographic data.

To utilize the SWAT model, input data from forecasted climate models are required. This data includes precipitation, temperature, solar radiation, wind speed, and relative humidity. In this research, due to the importance of high temperature in future climate changes and finally its effect on the amount of river flow, this fact has been given more attention. By running the SWAT model, it is possible to simulate the flow river and compare the resulting changes with historical the hydrological regime.

The mathematical method used for runoff simulation by the SWAT model scenarios is based on the water balance equation for each hydrological response unit (HRU) within the watershed. This equation follows:

(1) $$SW_{T}=SW_{0}+\sum_{i=1}^{t}\left(R_{i}-Q_{surf,i}-E_{i}-Q_{gw,i}-Q_{lat,i}-Q_{rev,i}\right)$$

Here, the final soil water content $SW_{T}$ is determined by various factors in the water balance equation. These factors include the initial soil water content $SW_{0}$, precipitation $R_{i}$, surface runoff $Q_{surf,i}$, evapotranspiration $E_{i}$, lateral flow $Q_{lat,i}$ , and return flow from irrigation or ponds $Q_{rev,i}$.

To forecast the river flow under climate changes using the SWAT model under RCP-SSP scenarios, the following steps must be undertaken.

1. Input data required for the SWAT model, including geological data, such as Digital Elevation Model (DEM) data, soil map data, and land use data, and watershed-specific climate data are preprocessed.
2. 3. Obtain future climate data (temperature) using GCMs models and downscale them to the basin scale.
3. Calibration and validation of the SWAT model are done by comparing it with observed river flow data from selected locations and periods.
4. Run the SWAT model using future climate data and geological data, as input, and get the forecasted flow data as output.
5. Changes in streamflow characteristics, including mean, variability, seasonality, and extremes, under different RCP-SSP scenarios are analyzed.

### 2.4 Hydroelectricity potential simulation

The potential impact of climate change on the hydroelectricity potential is significant due to the strong dependence of hydropower generation on the availability of water. This availability is influenced by various factors such as precipitation patterns, temperature, and evaporation rates. Climate change can alter these factors, leading to changes in river flow and subsequently affecting the potential for hydropower generation. For example, increased temperatures and changing precipitation patterns can change the timing and volume of snowmelt, impacting the seasonal distribution of runoff and water supply reliability for hydropower generation.

The athematical method used to calculate the potential for hydroelectricity is based on the potential energy of water, which is then converted into electrical energy. This theoretical power that can be harnessed from falling water, also known as hydropower, can be expressed using the following equation:

(2) $$P_{th}=\rho \cdot q\cdot g\cdot h$$

Here, the available power theoretically, denoted as $P_{th}$, is calculated using the formula where ρ represents the density of water (approximately 1000 kg/m³ for water), q represents the water flow rate in cubic meters per second (m³/s), g represents the acceleration due to gravity (9.81 m/s^2^), and h represents the falling height or head in meters.

However, in reality, the power that can actually be harnessed will be lower than the theoretical power due to energy losses in the system. To determine the practically available power, we need to consider the efficiency (μ) of the hydropower system, which takes into account losses in the turbines, generators, and other components.

(3) $$P_{a}=\mu \cdot \rho \cdot q\cdot g\cdot h$$

where $P_{a}$ shows the hydropower available (W).

Using this equation, the hydroelectricity potential of a site can be estimated by measuring or predicting the flow rate and head and taking into account the efficiency of the hydropower technology used. It should be emphasized that future changes in flow rate and head, which will impact the hydroelectricity potential calculations under different climate conditions, can be projected using climate change scenarios like RCP (Representative Concentration Pathways) and SSP (Shared Socioeconomic Pathways).

### 2.5 Thermoelectricity potential simulation

Thermoelectricity is a process that involves the conversion of heat energy into electrical energy via the use of thermoelectric materials. These materials can create a voltage difference when subjected to a temperature gradient. Thermo-Electric Generators (TEGs) use specific materials to produce electrical energy by converting waste heat or other heat sources. The efficacy of thermoelectricity is contingent upon many aspects, including the disparity in temperature, the efficiency and expense of the thermoelectric materials, and the availability and caliber of the heat source and cooling mechanism. The influence of climatic change on these variables may exhibit variability contingent upon the thermoelectric utilization's geographical context, typology, and magnitude.

For example, climate change has the potential to result in heightened occurrences and heightened severity of heat waves, thereby amplifying the disparity in temperature and augmenting the need for cooling measures. This phenomenon has supplementary prospects for the production and use of thermoelectric power. Nevertheless, climate change can potentially reduce both the quantity and the caliber of water resources, often used as a means of cooling for thermoelectric apparatus. As a result, the performance and dependability of such systems may be constrained. Moreover, climate change has the potential to impact the accessibility and economic viability of alternative energy resources, including fossil fuels, renewable energy, and nuclear power. Several variables may influence the competitiveness and appeal of thermoelectricity as an energy alternative.

The estimation of thermoelectric potential, taking into account the water supply for cooling systems, may be facilitated by using a mathematical approach. The approach used in this study is based on an equation that incorporates many factors.

(4) $$P_{T}=wa\cdot \rho \cdot q\cdot g\cdot h\cdot \eta$$

Here, the thermoelectric power output, denoted as $P_{T}$ , is determined by various factors. One of these factors is the water availability factor, represented by wa, which ranges between 0 and 1. The density of water, denoted as ρ, is approximately 1000 kg/m³. The water flow rate, q, is measured in cubic meters per second (m³/s). The acceleration due to gravity, g, is 9.81 m/s^2^. The falling height or head, h, is measured in meters (m). Lastly, the thermoelectric efficiency, η, is a value between 0 and 1. The water availability factor, μ, plays a crucial role in determining the fraction of water that can be utilized for cooling the thermoelectric device. It takes into account factors such as water scarcity, water quality, and environmental regulations. Estimating the water availability factor can be done through the use of hydrological models, water resources

The thermoelectric efficiency, denoted as η, quantifies the proportion of the total heat energy effectively transformed into electrical power by the thermoelectric device. This efficiency is determined by considering various factors such as the temperature difference, the Seebeck coefficient, the electrical resistivity, and the thermal conductivity of the thermoelectric material. To calculate the thermoelectric efficiency, the following equation can be utilized:

(5) $$\eta =\frac{T_{h}-T_{c}}{T_{h}+\frac{T_{c}}{ZT_{h}}}$$

Here, $T_{h}$ shows the hot side temperature (K), $T_{c}$ indicates the cold side temperature (K), and $ZT_{h}$ shows the figure of merit of the thermoelectric material (dimensionless). The formation of merit can be expressed as:

(6) $$ZT=\frac{S^{2}\sigma }{\kappa }T$$

Here, the Seebeck coefficient (S) is measured in volts per kelvin (V/K), the electrical conductivity (σ) is measured in siemens per meter (S/m), the thermal conductivity (κ) is measured in watts per meter per kelvin (W/m/K), and the average temperature (T) is measured (K).

The thermoelectricity potential of a location can be determined by assessing the water availability, water flow rate, head, hot and cold side temperatures, and the properties of the thermoelectric material. It is worth mentioning that climate change scenarios, like the ones outlined by RCP (Representative Concentration Pathways) and SSP (Shared Socioeconomic Pathways), can be employed to forecast alterations in these factors. These changes will subsequently impact the calculations of thermoelectricity potential under varying climate conditions.

### 2.6 Electricity demand and electricity prices simulation

#### 2.6.1 The echo state network

Lately, in RNNs, the dynamic reservoir has become a more popular choice than the hidden layer. As a result, the echo state network is now considered to be the newest version of RNN. Its comparative features consist of.

− Utilizing the reservoir's weight, which is randomly connected, is used as a component of processing data.
− The reservoir that has been received with inputs illustrates a feature area that is randomly produced.
− Weights of output are the only ones adapted during the training process, while other weights generally begin in a random initialization.
− A common method for learning the weight connections in Readout is linear regression.

The conventional ESN is illustrated in Fig. (3) and is composed of three primary steps: the readout, input, and reservoir layers. To improve the categorization accuracy, the input bias of a component is removed. The perception of a sparse, vast, and stochastically interconnected reservoir layer was offered. The complexity of the task heavily influences the number of elements present in ESN's reservoir, which can be pretty significant. Fig. (3) illustrates the structure of the Echo State Network (ESN), where the voluntary weight connections are represented by dotted lines.

**Fig. 3:** The framework of the Echo State Network.

The main way to obtain connection weights is by using a uniform distribution that is symmetrical around zero. In this study, a different ESN has been selected that has j inputs. In each iteration (q), $I\left(q\right)={\left[I_{1}\left(q\right),I_{2}\left(q\right),.\;.\;.,I_{S}\left(q\right)\right]}^{Q}$ inputs can be accomplished by the S neurons that are currently active. There are certain components in reservoir L, which are illustrated as $y\left(q\right)={\left[y_{1}\left(q\right),y_{2}\left(q\right),.\;.\;.,y_{L}\left(q\right)\right]}^{Q}$. Output K comprises certain elements that are represented as follows: ${\left[P_{1}\left(q\right),P_{2}\left(q\right),.\;.\;.,P_{K}\left(q\right)\right]}^{Q}$; Additionally, it has the capability to anticipate outcomes. It can be comprehended that the updated equation of the reservoir is indicated as follows:

(7) $$y\left(q\right)=b\left(W^{in}I\left(q\right)+W^{r}y\left(q-1\right)+W^{back}P\left(q-1\right)\right)$$

Moreover, the formula for output has also been provided as follows:

(8) $$P\left(q\right)=v\left(W^{inout}I\left(q\right)+W^{out}y\left(q\right)+W^{outout}P\left(q-1\right)\right)$$

Here, b indicates the input of the AF (activation function), and v illustrates the output of the AF. $W^{in}\left(S\times L\right)$ defines the input of the weight's matrix link, which is between the inputs and the reservoir. $W^{r}\;\left(L\times L\right)$ represents the connection weight of the reservoir. The weights of the feedback that are voluntary and exist between the reservoir and the output are depicted by $W^{back}\;\left(K\times L\right)$. A few optional links are also available, and $W^{inout}\left(S\times K\right)$ illustrates certain weights between the input and output. $W^{outout}\;\left(K\times K\right)$ is utilized to represent the weights of the output cycle, while $W^{biasout}\left(1\times K\right)$ demonstrates the bias and output weights. It was previously mentioned that only the output weights need to be trained. However, the connections between the existing weights are usually created randomly and tend to remain stable throughout the ESN training procedure. After determining the total weight's links to output by $W^{outGen}$, some adjustments are applied using the following formulation:

(9) $$P\left(q\right)=v\left(W^{outGen}\left[I\left(q\right);y\left(q\right);P\left(q-1\right)\right]\right)$$

Here, P(q) represents matrix concatenation. Discovering $W^{outGen}$ is the primary aim of this training procedure. It is possible to modify the formulation by assuming that the variable v can be inverted in the earlier formulation:

(10) $$X=W^{outGen}\left[I\left(q\right)y\left(q\right);P\left(q-1\right)\right]$$

Here, X approximately is equivalent to $v^{-1}P\left(q\right)$. Using the method of the least squares regression, the output weight is computed. The aim is to reduce the distinction between the network's actual output and its anticipated output.

Regarding the important feature of the echo's state network, the Echo State Property (ESP) indicates that the impact of earlier circumstances and initial inputs on future requirements should decrease over time, with no necessary improvements. Observations from practical applications have shown that the ESP remains valid as the weight of the reservoir increases. Consequently, the maximum amount of eigenvalue $W^{r}$, which is considered to be less than one, results in an SR (Spectral Radius). Some research suggests that external stimuli may affect the ESP of ESN. In specific input conditions, the ESN can accomplish ESP even when the SR is greater than one.

#### 2.6.2 Modified Snow Leopard Optimization Algorithm

The snow leopard is featured in the introduction, followed by the introduction of a recently developed optimization algorithm called the Snow Leopard Optimization (SLO) algorithm. The algorithm's creation was influenced by the snow leopard's natural activities and behavior. The passage also presents a suggestion for a numerical model of SLO to be utilized in solving optimization problems.

(A) Snow Leopard

Panthera uncia, also known as snow leopard, can be found in the elevated mountains of Central and South Asia. These creatures are difficult to spot and inhabit in regions with high altitudes, ranging from 3000 to 4500 m. They can be found in several areas like the Himalayas, western China, southern Siberia, the Tibetan Plateau, eastern Afghanistan, and Mongolia.

The fur color of snow leopards can range from white to gray, and they have black spots on their neck and head. The snow leopards’ back and sides feature longer rosettes, and their tail is covered with hair. They have a white underbelly, as well as gray or light green eyes, large nasal cavities, a short snout, and a rounded forehead. The dense fur of snow leopards consists of hairs whose length is between 5 and 12 cm. Compared to other members of the Panthera family, this animal is characterized by short legs and a strong body. It is smaller than its relatives and can reach a maximum height of 56 cm when it stands up. Its body length is in the range of 75–150 cm. Its tail can be in the range of 80–105 cm. The weight of the animal can range from 22 to 55 kg, with some bigger males weighing up to 75 kg and smaller females weighing less than 25 kg, depending on the candidate. The animal is distinguished from other members of the Panthera species by its slim, 28.6 mm long canine teeth.

Snow leopards have different behaviors that include their social interactions, ways of transportation, hunting techniques, reproductive processes, and mortality rates. The suggested Snow Leopard Optimization Algorithm design has four ideal behaviors that are commonly observed in the life of snow leopards, with the aim of emulating their natural tendencies. Snow leopards use breeding as their primary method for mating. This process includes two members of the population that come together to produce offspring that could potentially enhance the algorithm's capacity to reach the best locations. Optimizing the algorithm to find the best areas for catching prey can be improved by illustrating the evaluation of snow leopard hunting. This is the third methodology employed for this purpose.

To enhance the analysis of the solution space and effectively navigate through the optimal local areas, it is preferable to demonstrate the zigzag movements of snow leopards while they move and pursue one another. This can be completed by illustrating their travel paths and motion, which is the third approach.

The fourth method is a fatal outcome, which demonstrates how the incapability of snow leopards leads to the removal of possible solutions and the exclusion of inappropriate members from the solution space of the algorithm. This also guarantees a consistent population of the algorithm during its repetitions.

(B) Mathematical Modeling

The Snow Leopard Optimization Algorithm suggests that a snow leopard can be considered as an algorithm population member and performs the role of a search agent. To identify the population members, the population-based optimization algorithms utilize a population matrix. The matrix consists of rows and columns that represent the number of members and variables in the optimization problem, respectively. The matrix of the population is defined by a definite formulation:

(11) $$A={\left[\begin{array}{c} A_{1}\\ \vdots \\ \begin{array}{c} A_{i}\\ \begin{array}{c} \vdots \\ A_{N} \end{array} \end{array} \end{array}\right]}_{N\times m}=\left[\begin{array}{ccc} A_{1,1} & \cdots & \begin{array}{cc} A_{1,d} & \begin{array}{cc} \cdots & A_{1,m} \end{array} \end{array}\\ \vdots & \ddots & \begin{array}{cc} \vdots & \begin{array}{cc} \ddots & \vdots \end{array} \end{array}\\ \begin{array}{c} A_{i,1}\\ \begin{array}{c} \vdots \\ A_{N,1} \end{array} \end{array} & \begin{array}{c} \cdots \\ \begin{array}{c} \ddots \\ \cdots \end{array} \end{array} & \begin{array}{cc} \begin{array}{c} A_{i,d}\\ \begin{array}{c} \vdots \\ A_{N,d} \end{array} \end{array} & \begin{array}{cc} \begin{array}{c} \cdots \\ \begin{array}{c} \ddots \\ \cdots \end{array} \end{array} & \begin{array}{c} A_{\left(i,m\right)}\\ \begin{array}{c} \vdots \\ A_{N,m} \end{array} \end{array} \end{array} \end{array} \end{array}\right]$$

Here, A illustrates the snow leopards' population, and $A_{i}$ demonstrates the $i^{th}$ snow leopard. The quantity of the problem variable proposed by the $i^{th}$ ,snow leopard is demonstrated by $A_{i}$ for the $d^{th}$ problem. Cap N is utilized in the population algorithm to represent the number of snow leopards, while m signifies the number of problem variables. The problem-solving space is defined by the situation of each snow leopard member in the population, which determines the values of the problem variables. Each snow leopard's cost function can be computed based on a specific value. The formulation given determines the vector that represents the cost value:

(12) $$X={\left[\begin{array}{c} X_{1}\\ \vdots \\ \begin{array}{c} X_{i}\\ \begin{array}{c} \vdots \\ X_{N} \end{array} \end{array} \end{array}\right]}_{N\times 1}=\left[\begin{array}{c} X\left(A_{1}\right)\\ \vdots \\ \begin{array}{c} X\left(A_{i}\right)\\ \begin{array}{c} \vdots \\ X\left(A_{N}\right) \end{array} \end{array} \end{array}\right]$$

Here, X illustrates the vector of cost values. $X_{i}$ demonstrates the number of cost values for a specific problem on the basis of the $i^{th}$ snow leopard.

In the Snow Leopard Optimization Algorithm, the renewal of the population is accomplished by following the natural behaviors of snow leopards that consist of four phases: movement, hunting, breeding, and death. These phases are expressed mathematically, and the corresponding natural behaviors are explained in the following parts.

##### 2.6.2.1 Phase 1: Movement

Snow leopards, like other kinds of cats, use scent markings to signal their location and travel routes. They usually create these marks by scratching the ground with their back legs before leaving behind feces or urine. Snow leopards are known for their unique zigzag pattern of movement, which enables them to follow each other naturally. The current phase of the proposed SLO Snow Leopard Optimization Algorithm is defined using particular formulas:

(13) $$\begin{array}{c} A_{i,d}^{F1}=A_{i,d}+r\times \left(A_{k,d}-1\times A_{i,d}\right)\times sign\left(\;X_{i}-X_{k}\right)\;k\in 1,2,3,4,\ldots .,N\\ d=1,2,3,4,\ldots .,m \end{array}$$

(14) $$A_{i}=\left\{ \begin{array}{c} A_{i}^{F1},X_{i}^{F1}\;<X_{i}\\ A_{i} \end{array}\right.$$

(15) I=round(1+r)

Here, the updated value of the $d^{th}$ problem variable that is obtained by the $i^{th}$ snow leopard in the initial phase is demonstrated by $A_{i,d}^{F1}$, and r is a random number that ranges between 0 and 1. The guidance of the $i^{th}$ snow leopard is provided by a particular snow leopard denoted by the row number k in the $d^{th}$ dimension. ${\;A}_{i}^{F1}$ represents the updated location of the $i^{th}$ individual after the initial phase, and its cost value is illustrated by $X_{i}^{F1}$.

##### 2.6.2.2 Phase 2:

In the second phase of renewal, the snow leopard employs its techniques for hunting and assaulting its target. Researchers have observed in Hemis National Park that the snow leopard utilizes rocky cliffs to cover itself when it is close to its target. The snow leopard gets closer to its prey from a distance of 40 m, then walks 15 m towards it, and then runs 25 m with great force. Finally, the snow leopard bites its prey's neck to attack it and capture it successfully.

The method in which snow leopards hunt is determined by two formulas, namely Eq. (14) and Eq. (15). Eq. (14) specifies the location of the prey relative to each snow leopard, while Eq. (15) describes the approach that a snow leopard employs when pursuing its target. In this part, the hunting technique of snow leopards is explained. To demonstrate the movement, a cap X is utilized in Eq. (15). According to the equation, the snow leopards take a stride that covers 0.375 percent of the distance and then run the remaining 0.625 percent of the distance to reach and capture their prey. The parameter in Eq. (15) illustrates the ratio of the distance that the snow leopard strides towards its prey.

The Snow Leopard Optimization Algorithm includes a variable that indicates how far a snow leopard can stride compared to the distance of its prey. Based on the instructions for reproducing the Snow Leopard Optimization Algorithm, this variable is fixed at a value of 0.375. Eq. (16) is a model of the snow leopard's behavior following a successful hunt:

(16) $$f_{i,d}=a_{i,d},d=1,2,3,4,\ldots .m$$

(17) $$A_{i,d}^{F2}=A_{i.d}+r\times \left(\left(f_{i,d}-A_{i,d}\right)\times F+\left(F_{i,d}-2\times A_{i,d}\right)\times \left(1-F\right)\right)\times sign\left(\;X_{i}-X_{f}\right)$$

(18) $$A_{i}=\left\{ \begin{array}{c} A_{i}^{F2},X_{i}^{F2}<\;P_{i}\\ A_{i} \end{array}\right.$$

$f_{i,d}$ end subscript illustrates the value of the situation of the prey in the $d^{th}$ dimension. The cost value based on the situation of the prey is illustrated by $X_{f}$. The value $X_{i,d}^{F2}$ demonstrates the new amount obtained by the $i^{th}$ snow leopard based on the second phase for the $d^{th}$ dimension and the related cost value is demonstrated by $X_{i}^{F2}$.

##### 2.6.2.3 Phase 3: Breeding

The algorithm increases its population by half for every new member based on the natural breeding habits of snow leopards. Snow leopards breed by pairing two individuals, leading to the birth of a cub. The breeding procedure of the snow leopard is mathematically evaluated by applying the mentioned concepts in the given formula:

(19) $$B=\frac{a_{1}+a_{N-l+1}}{2},l=1,2,3,4,\ldots ‥\frac{N}{2}$$

The value $B_{l}$ is the $l^{th}$ cub that was born from a female and a male snow leopard.

##### 2.6.2.4 Phase 4: Death

Living organisms always face the risk of death. Despite the fact that breeding programs have been implemented to raise the population of snow leopards, their numbers remain constant due to mortality and other issues. The Snow Leopard Optimization Algorithm suggests that an equal number of snow leopard cubs will be dead during every breeding cycle. According to the principle of snow leopard death in the Snow Leopard Optimization Algorithm, snow leopards with a low-cost value are more likely to die. Additionally, having a weak cost value also endangers the lives of newborn cubs.

(C) Modified Snow Leopard Optimization algorithm

Tuning of variable: Modify the random number range (r) includes utilizing a dynamic update regulation that depends on the population's effectiveness, as demonstrated in the example below:

(20) $$r_{i+1}=r_{i}+c\times \left(1-e^{k\times fitness_{diff}}\right)$$

Here, the fundamental range value is demonstrated by $r_{i}$, the difference in fitness levels between the best and the worst candidate is illustrated by $fitness_{diff}$, a consistent learning rate is demonstrated by c, and a scaling element is demonstrated by k.

To modify the ratio of stride to prey distance, a straightforward method involves implementing the parameter p that manages the size of the stride. The method of updating can be defined as follows:

(21) $$A_{i}^{F1}=A_{i}^{F1}+r\times \left(A_{k,d}-A_{i,d}\right)\times sign\left(X_{i}-X_{k}\right)\times p$$

The implementation of the crowding technique has been done in order to preserve diversity. The crowding distance technique is one of the simple approaches to achieve this goal, which measures the distance between solutions in the objective space. To express the updated rule formulation, the following equation has been utilized:

(22) $$fitness_{i+1}=fitness_{i}+\alpha \times crowding_{distance_{i}}$$

where,

(23) $$crowding_{distance_{i}}=sum\left(dist\left(A_{i},A_{j}\right)\;for\;j\;in\;population\;if\;i\neq j\right)$$

The variable α is a crowding element, and $fitness_{i}$ is the novel fitness value for the candidate $A_{i}$, and $dist\left(A_{i},A_{j}\right)$ is the distance of Euclidean between the vectors of $A_{i}$ and $A_{j}$.

The chosen set parameters for the Modified Snow Leopard Optimization algorithm are as follows: the stochastic range (r) is set to rand (0,1), the learning rate (c) is set to 0.01, the scaling factor (k) is set to 0.1, the stride proportion (p) is set to 0.5, and the crowding factor (α) is set to 0.5.

(D) Algorithm authentication

In this part, we examined the Modified Snow Leopard Optimization Algorithm against other advanced algorithms such as Pelican Optimization Algorithm (POA) [23], Sine Cosine Algorithm (SCA) [24], Gravitational Search Algorithm (GSA) [25], Squirrel Search Algorithm (SSA) [26], and Multi-Verse Optimizer (MVO) [27], Biogeography-Based Optimizer (BBO) [28]. Assessing the performance of algorithms on shifted classic benchmark functions and the CEC2017 benchmark functions was the primary objective of this investigation.

These benchmark functions are widely recognized in the optimization field as standardized and established test cases. This allows for an equitable comparison between various algorithms. In order to evaluate the effectiveness of the algorithms, we employed performance measurements standard deviation (STD). These measurements offer valuable information about the algorithm's capacity to consistently discover solutions and its general precision in achieving the best solution. The effectiveness of algorithms can be measured by testing their performance on problem cases where the best solution is moved from the origin and comparing the outcomes of two versions.

#### 2.6.3 Optimizing the ESN based on MSLO for accurate estimation

The optimization of the Echo State Network (ESN) through the Modified Snow Leopard Optimization Algorithm is designed to increase the accuracy of estimation within the network. By utilizing this algorithm, the ESN goes through a refinement and tuning process to enhance its performance in data prediction and analysis. Drawing inspiration from the behavior of snow leopards in the wild, the Modified Snow Leopard Optimization Algorithm introduces specific rules and mechanisms to iteratively adjust the parameters and structure of the ESN iteratively, resulting in more precise and reliable estimations. This optimization strategy aims to fine-tune the ESN's configuration to capture better the underlying patterns and dynamics of the processed data, thereby improving its predictive capabilities and overall efficiency across various applications.

The Modified Snow Leopard Optimization Algorithm has the potential to enhance the performance of Echo State Network (ESN) and improve the accuracy of estimations in diverse applications. Below is a brief summary of the optimization process.

− Initialization: The ESN parameters, including reservoir size, spectral radius, and input scaling, are set at the same time as the parameters of the Snow Leopard Optimization Algorithm.
− Fitness Function: A fitness function has been established to assess the effectiveness of the ESN model according to particular criteria, including prediction accuracy and error metrics.
− Population Evolution: The Modified Snow Leopard Optimization Algorithm continuously adjusts the solution population by emulating the hunting tactics of snow leopards. This method combines exploration and exploitation to find the best set of ESN parameters.
− Parameter Update: The ESN parameters, such as reservoir weights, input weights, and bias terms, are modified by the algorithm according to fitness evaluations in order to enhance the model's accuracy.
− Convergence: The optimization procedure persists until a termination condition is satisfied, such as achieving a specified number of iterations or attaining a desirable level of performance.
− Performance Evaluation: The accuracy of estimating the desired output is assessed by evaluating the optimized ESN model using validation data. To measure the improvement achieved through the utilization of the Modified Snow Leopard Optimization Algorithm, the performance metrics are compared with baseline models or other optimization techniques.

Through the utilization of the Modified Snow Leopard Optimization Algorithm to enhance Echo State Networks, researchers can adjust the ESN parameters in order to improve the precision and predictive capabilities of the model across a range of applications, including time-series forecasting, pattern recognition, and signal processing. The combination of ESNs and nature-inspired optimization algorithms has the potential to result in more reliable and effective estimation methods in intricate situations.

#### 2.6.4 Training the echo state network based on the MSLO

The confirmation data's Mean Squared Error (MSE) is utilized as the cost function in the current investigation. A portion of the training data is reserved for verifying every agent. Then, the parameters are selected, and the Echo State Network is trained. The cost function of the agent on the confirmation data is determined by the mean squared error of the echo state network. The cost function of MSE can be represented by the following formula. Each column's input weight matrix is scaled by normalizing it with the highest value, which is then normalized to a parameter. The normalization of the reservoir matrix in relation to the MSLO involves dividing it by the maximum eigenvalue and then normalizing it to the Spectral Radius. This is performed before its normalization to the Spectral Radius.

(24) $$MSE=\frac{1}{n}\sum_{i=1}^{n}{\left(P_{i}-\hat{P_{i}}\right)}^{2}$$

Here, the expected output is demonstrated by P, and the actual output is illustrated by $\hat{P}$.

### 2.7 Forecasting electricity demand by optimal ENS

Electric energy is an essential driving force for economic development, while the accuracy of demand Electric energy plays a crucial role in facilitating economic growth, while the precision of demand prediction is a significant determinant of the effectiveness of productivity planning. Due to this rationale, it is essential for energy analysts to possess a framework that aids in selecting the most suitable forecasting methodologies, hence ensuring the provision of precise projections about power consumption patterns. Numerous methods exist to forecast future power consumption. The power consumption assessment is crucial in light of the rising electricity demand. The growing worldwide demand for power necessitates the development of sophisticated forecasting techniques and algorithms. Accurately predicting power consumption over an extended period is fundamental to formulating energy investment strategies and is essential for governments in emerging nations. The act of overestimating demand may lead to the presence of excessive idle capacity, resulting in the inefficient allocation of financial resources. Conversely, underestimating consumption may lead to elevated operating expenses for the energy supply and the probable occurrence of power outages. Hence, ensuring precise modeling of power usage is of utmost importance to prevent expensive errors.

To forecast electricity consumption with Echo State Networks (ESN), it is necessary to do the following sequential procedures:

The power demand data should undergo preprocessing techniques, including normalization, smoothing, and outlier removal, to prepare it for input into an Echo State Network (ESN) model.

The selection of hyperparameters for the Echo State Network (ESN) involves determining values for many parameters, including the reservoir size, spectral radius, input scaling, leakage rate, and regularization parameter. The performance and stability of the Echo State Network (ESN) are influenced by these hyperparameters, which techniques like cross-validation or grid search may optimize.

The reservoir matrix $W_{res}$ , input matrix $W_{in}$ , and feedback matrix $W_{fb}$ are initialized randomly, according to specific distribution and sparsity requirements. To maintain the echo state property, the reservoir matrix needs to possess a spectral radius, denoting the maximum absolute eigenvalue, that is less than unity. This condition guarantees that the reservoir state effectively diminishes the influence of its prior values as time progresses.

The Echo State Network (ESN) is trained on the power demand data via Input sequence u(n) fed into the reservoir. At each time step n, the reservoir position x(n) is collected. The equation provided is used to update the reservoir position

(25) $$x\left(n\right)=\left(1-\alpha \right)x\left(n-1\right)+\alpha \;\tanh\;\left(W_{in}u\left(n\right)+W_{res}x\left(n-1\right)+W_{fb}y\left(n-1\right)\right)$$

Here, the leakage value, denoted by α, and the output feedback, represented by y(n-1), are essential factors in the context. The output layer, Wout, is determined through linear regression techniques, such as ridge regression or least squares. This process involves utilizing the reservoir states and the target sequence, y(n), that have been gathered.

(26) $$W_{out}=YX^{T}{\left(XX^{T}+\beta I\right)}^{-1}$$

Here, the regularization parameter, denoted as β, is accompanied by the identity matrix, represented as I.

The experimental evaluation of the Echo State Network (ESN) involves assessing its performance on novel power demand data. This is achieved by providing the input sequence u(n) to the reservoir and calculating the network output y(n) at each time step n.

The performance of the ESN may be assessed by the use of many measures, including mean absolute error (MAE), root mean squared error (RMSE), or mean fundamental percentage error (MAPE). These metrics quantify the disparity between the network output, denoted as y(n), and the actual power demand, represented as d(n)..

(27) $$\text{MAE}=\frac{1}{N}\sum_{n=1}^{N}|y\left(n\right)-d\left(n\right)|$$

(28) $$\text{RMSE}=\sqrt{\frac{1}{N}\sum_{n=1}^{N}{\left(y\left(n\right)-d\left(n\right)\right)}^{2}}$$

(29) $$\text{MAPE}=\frac{1}{N}\sum_{n=1}^{N}\frac{|y\left(n\right)-d\left(n\right)|}{d\left(n\right)}$$

Here, N shows the time stages number.

Several discussions have been conducted regarding the use of Echo State Networks (ESN) for power demand prediction. One notable advantage of ESN is its ability to capture the nonlinear and nonstationary characteristics of power demand data, enabling it to generate accurate and robust forecasts for both short-term and long-term horizons. Additionally, ESN can be effectively combined with other techniques, such as metaheuristic algorithms, to enhance its performance and generalization capabilities further.

### 2.8 Forecasting electricity price by optimal ENS

The steps for price forecasting using ESN are similar to those for power demand forecasting but with some adjustments. Here are the key differences.

1. Input: The ESN input consists of historical price data for the desired electricity demand for price forecasting.
2. Output: The output of ESN in price prediction is the expected future price of the desired electricity. Depending on the specific application and data availability, a forecast horizon can be selected, such as one day ahead, one week ahead, or one month ahead. Additionally, depending on the range and distribution of the output, you can use different output activation functions such as sigmoid.
3. Evaluation: ESN's price forecasting evaluation revolves around the forecasts' accuracy and profitability. To evaluate the accuracy of projections, you can use measures such as Mean Absolute Error (MAE), Root Mean Square Error (RMSE), or Mean Percent Fundamental Error (MAPE).

## 3 Results

### 3.1 Temperature and flow river forecasting under climate changes

Fig. (4)displays the predicted fluctuations in the average monthly temperature of Yunnan, considering various socio-economic-climate scenarios. These projections are derived from the 2000–2023 baseline data to forecast temperature from 2024 to 2854.

**Fig. 4:** The forecasted fluctuations of temperature under SSP-RCPs.

Temperature projections by CanESM5 show that global surface temperatures will increase under all scenarios, but the magnitude and pattern of warming will vary by scenario. For example, in the low-emissions scenario SSP1-2.6, the global mean temperature by 2053 will increase by about 0.57 °C relative to pre-industrial levels, while in the high-emissions scenario SSP5-8.5, the global mean temperature by 2053 will be about It increases by 1.65 °C. The SSP5-8.5 scenario will have the highest and most constant increase, while the SSP1-2.6 method will have the lowest and most variable increase. The SSP2-4.5 scenario will have moderate growth. Future temperature changes in winter and spring will be more significant than in summer and autumn. Due to the reduction of snow cover and increased heat absorption by greenhouse gases, the temperature increase changes in winter and spring are expected to be more than in summer and autumn. However, the summer season will have the highest temperature increase in July and December will have the lowest temperature. These temperature changes can significantly affect the availability of water needed to generate electricity in the electrical system, and the performance of the cooling systems in the thermoelectric station.

The simulation of river flow in Yunnan under different climate scenarios has been conducted using the SWAT model in this research. The Xiangjiaba Station, located in the lower part of the Jinsha River, has reported a yearly runoff of 83.25 billion m³ in 2023. The expected changes in monthly runoff (in million m³) at the Xiangjiaba station under various climate scenarios from 2024 to 2054 are depicted in Fig. 5.

**Fig. 5:** The runoff forecasting under SSPs-RCPs.

The results showed that Yunnan's annual runoff will decrease compared to the period of 2000–2023 by the end of the 2053. The decrease in runoff will be more evident in the dry season than in the wet season.

### 3.2 The thermoelectric and hydropower potential forecasting under climate change

The hydropower potential at Xiangjiaba has been affected by different climate scenarios, as shown in the Fig. (6).

**Fig. 6:** The hydropower potential forecasting.

In the SSP1-RCP2.6 scenario, a reduction of around 0.56 GW in hydropower capacity was observed. Similarly, the SSP2-RCP4.5 scenario resulted in a decrease of about 0.88 GW. However, the most notable impact was witnessed under the pessimistic SSP5-RCP8.5 scenario, where a remarkable reduction of approximately 1.65 GW occurred. These findings highlight the significant and concerning effect on hydropower capacity under the SSP5-RCP8.5 scenario, emphasizing the urgent need for proactive measures and sustainable strategies to mitigate these adverse consequences.

Fig. (7)exhibits the monthly capacity (MW) of the Diandong Power Station, a coal-fired thermal power plant situated in Yunnan. With a formidable capability of 2.4 GW, this thermoelectric facility serves as a substantial energy provider within the region.

**Fig. 7:** Thermoelectricity potential under SSP-RCPs.

These findings highlight the sensitivity of Diandong power plants' potential to climate change. The graph depicts the month-to-month variability of power potential across various scenarios. Notably, the highest values are observed in July and August, while the lowest values are evident in December and January. This suggests that during the summer season, when there is increased rainfall, the limitation of water supply for cooling systems is less than in dry months, resulting in better production. However, as global warming progresses, there is a noticeable decline in power potential, which will lead to reduced performance in thermoelectricity in the future.

### 3.3 Potential consequences of factors affecting the decrease in hydropower

− Factors Contributing to decline in hydropower potential:

The notable decline in hydropower potential across various climate scenarios, especially in the SSP5-RCP8.5 scenario, can be attributed to a number of important factors:

Limited Water Availability: Changes in rainfall patterns caused by climate change and higher rates of evaporation can result in a decrease in water availability in rivers and reservoirs, affecting the overall water supply for hydropower production.

Changed Flow Patterns: Fluctuations in river flow patterns such as flow reductions and seasonal changes, have the potential to impact the effectiveness and dependability of hydropower plants, ultimately diminishing their capacity to produce electricity.

Glacial Melting: In situations such as SSP5-RCP8.5, where there is a notable increase in temperatures, the rapid melting of glaciers may initially boost water availability. However, in the long run, it can result in reduced water flow, impacting the efficiency of hydropower facilities.

Extreme Weather Events: The increased occurrence and severity of extreme weather events, such as droughts and floods, have the potential to interrupt hydropower generation and infrastructure, leading to a negative impact on hydropower generation.

− The implications and potential consequences of these reductions:

The implications of the notable reduction in hydropower potential across diverse climate scenarios, notably in SSP5-RCP8.5, are extensive and can lead to several ramifications.

Energy Security Concerns: Energy security concerns can arise from a decline in hydropower potential, as the reduced use of hydropower for electricity generation could lead to an increased reliance on less sustainable or environmentally friendly energy sources.

Economic Impact: The reduction in hydropower potential can lead to augmented expenses in generating electricity, thereby resulting in escalated electricity prices for consumers. This can have noteworthy financial ramifications, impacting industries and households that rely on cost-effective electricity.

Environmental Effects: Alterations in hydroelectric power production have the potential to impact nearby ecosystems and biodiversity. Variations in the flow patterns of rivers may lead to disturbances in aquatic habitats and the migration behaviors of marine species.

Adaptation Challenges: To effectively adapt to the diminishing potential of hydropower in the wake of changing climate scenarios, significant financial resources must be allocated towards alternative energy sources and the upgrading of infrastructure. This, however, presents a set of complex challenges for energy management and the formulation of appropriate policy decisions.

### 3.4 Impact climate changes on electricity demand and electricity price

In this section to forecast electricity demand and electricity price the optimized ENS model has been used. To validate suggested model, it has been compared with other metaheuristics model. The outcomes are evaluated through a statistical test applied to the CEC2017 benchmark functions, as identified in Fig. (8).

**Fig. 8:** Algorithm performance based on CEC2017 benchmark functions.

Valuable insights into the individual strengths and weaknesses of advanced algorithms can be obtained by analyzing the effectiveness of the Modified Snow Leopard Optimization Algorithm and comparing it with other algorithms on standard functions. The purpose of this analysis is to assess how well Modified Snow Leopard Optimization performs in solving optimization problems, significantly when the best solutions are displaced from the origin. The outcomes demonstrate that the suggested MSLO algorithm is highly effective and can optimize the arrangement of ENS by working on its loss function to offer an ENS-MSLO.

Monthly electricity demand has been forecasted by ENS-MSLO model. The monthly electricity demand in Yunnan from January to December (GWh) forecasting results has been shown in Fig. (9).

**Fig. 9:** The monthly electricity demand forecasting.

Yunnan province in southern China encounters a range of obstacles due to the fluctuating electricity demand it experiences throughout the year. Despite having ample water energy resources, these resources can only meet the market's needs during the wet months, resulting in a deficit during the dry winter months. As a result, the demand for electricity in Yunnan reaches its peak during the dry winter months and diminishes when hydropower is plentiful. The fluctuation in electricity consumption is a result of the province's utilization of various energy sources throughout different times of the year. Despite having abundant water energy resources, the region mainly relies on them in the warmer seasons of summer and spring. In contrast, coal-fired power plants are essential for fulfilling energy needs during the colder, drier winter months.

Yunnan's electricity demand experiences seasonal fluctuations, which are influenced by various factors. In the summer and spring seasons, the region predominantly depends on water energy resources owing to the copious rainfall and snowmelt. This abundance of water contributes to increased availability of hydropower. Consequently, rivers and reservoirs witness higher water levels during this period, thereby enhancing the efficiency and cost-effectiveness of hydropower generation.

During the dry winter months, the decline in water levels results in a decrease in hydropower generation capacity. In response to this issue and to fulfill the high electricity demand during this period, Yunnan province has resorted to utilizing coal-fired power plants. Coal-fired plants provide a dependable energy source that can function consistently regardless of weather conditions or water availability.

The strategic utilization of diverse energy sources in different seasons is aimed at optimizing energy generation according to the availability of resources and demand trends. By effectively managing the use of water energy resources and coal-fired power plants throughout the year, Yunnan can guarantee a more stable and reliable electricity supply to cater to the varying requirements of its population and industries.

The findings indicate that the projected electricity demand in Yunnan province will experience a notable increase in the future. This rise in demand can be attributed to various factors outlined in the scenarios SSP1-RCP2.6 and SSP5-RCP8.5. In the more optimistic scenario SSP1-RCP2.6, which focuses on sustainable development and reduced greenhouse gas emissions, the estimated increase in electricity demand is approximately 3.37 GWh. This growth can be attributed to factors such as population growth, economic development, and the adoption of energy-efficient technologies. As the population and economy expand, there will be a steady increase in the demand for electricity in the residential, commercial, and industrial sectors. Additionally, the transition towards cleaner and more sustainable energy sources will also contribute to the rise in electricity demand as more renewable energy projects are implemented.

On the other hand, the worst-case scenario SSP5-RCP8.5, characterized by high greenhouse gas emissions and unsustainable development, projects a much higher increase in electricity demand, reaching up to 13.1 GWh. This significant rise can be attributed to accelerated industrialization, urbanization, and a greater reliance on energy-intensive activities. The rapid expansion of industries and manufacturing sectors will lead to a surge in electricity consumption for production processes and machinery. Furthermore, increased urbanization will result in a higher demand for residential electricity for heating, cooling, lighting, and appliances. Given these projections, it is evident that there will be a substantial increase in future energy needs in Yunnan province. Therefore, careful planning and infrastructure development are crucial to meet the rising demand and ensure a reliable and sustainable energy supply for the region.

Electricity prices may vary across regions and sectors depending on electricity supply and demand, the availability and cost of different energy sources, the level and type of carbon pricing, and the degree of market integration and competition. The electricity price rate forecasting based on optimal ENS under socio-economic scenarios has been provide in Fig. (10).

**Fig. 10:** The electricity price forecasting.

This segment focuses on analyzing the influence of drought on electricity pricing in Yunnan, with a forecasted 2.98 % escalation in prices under the pessimistic scenario (SSP5-RCP8.5). This surge is attributed to factors like increased demand, reduced water supply for hydroelectric plants, and potential costs associated with carbon emissions. In contrast, the optimistic scenario (SSP1-RCP2.6) predicts a 1.7 % increase, possibly due to enhanced water management, the utilization of alternative energy sources, and the implementation of energy efficiency strategies.

In the ideal scenario (SSP1-RCP2.6), there is an expected moderate increase of about 0.34 %. This is made possible through the adoption of advanced energy management practices, diversification, and resilience to environmental and economic uncertainties. This outcome indicates a rising trend towards the end of the year, with the worst-case scenario reaching its peak. Conversely, the ideal system experiences a gradual price hike. The research concludes that the system's flexibility, diversity, and efficient practices help to moderate price increases, even in challenging circumstances.

The anticipated rise in prices across all situations is a result of the energy crisis caused by the drought that is affecting the water supply for hydroelectric plants in Yunnan. This has a direct impact on the generation of electricity from these renewable sources, resulting in a decrease in supply and subsequent increases in prices. The comparatively smaller increase in the best-case scenario could be attributed to successful measures taken to mitigate the crisis or the utilization of alternative energy sources that counterbalance its effects. This could potentially involve the implementation of better storage solutions, a more diverse energy mix, or the adoption of improved energy management practices.

In addition, the optimal scenario probably includes greater resilience in the energy infrastructure or proactive crisis management measures, which can restrict price escalation. Enhanced regulatory frameworks, robust market mechanisms, and efficient demand-side management practices may also assist in lessening the impact on electricity prices in this situation. Essentially, the marginal 0.34 % increase in the ideal scenario underscores the significance of strategic planning, resilience, and adaptability in mitigating the effects of the energy crisis on electricity prices.

## 4 Conclusion

The study examines the impact of water resource limitations on thermoelectric and hydroelectric stations' potential, electricity demand, and price. General Circulation Models (GCMs) and Soil and Water Assessment Tools (SWAT) are utilized to predict future temperature trends and river flow patterns. An optimized echo mode network (ESN) based on the Modified Snow Leopard Algorithm (MSLO) are used for optimizing ESN to estimate electricity demand and price accurately. The study shows a significant decrease in hydropower potential under different climate scenarios, with the most significant impact in the pessimistic SSP5-RCP8.5 scenario. The reductions are estimated to be around 0.56 GW for SSP1-RCP2.6, 0.88 GW for SSP2-RCP4.5, and 1.65 GW for SSP5-RCP8.5. The electricity demand is predicted to rise significantly, with an estimated increase of 3.37 GWh in the best-case scenario and 13.1 GWh in the worst-case scenario. The study predicts an increase in electricity prices across all three plans, with the ideal system expected to be less severe by 0.34 %. The pessimistic scenario predicts a 2.98 % average increase in the coming years, while the optimistic scenario predicts a moderate increase of 1.7 %.

The General Circulation Models (GCMs) have certain limitations due to their reliance on simplified representations of intricate climate processes, and their precision is contingent upon the availability of data. Furthermore, the study primarily emphasizes the significance of hydropower and thermoelectric systems, failing to adequately explore the potential of other renewable energy sources and their intricate relationships with water resources. Moreover, the economic impact assessment solely focuses on electricity prices, disregarding wider economic ramifications such as unemployment and industrial transformations stemming from shifts in energy production.

Future investigations should concentrate on the integration of modeling, strategies for adapting to climate change, approaches that span multiple sectors, support for policies and decisions, innovative pricing mechanisms, engagement with stakeholders, and technological advancements. These efforts should involve the development of models that take into account water availability, energy demand, and economic factors, the exploration of adaptive strategies for hydropower and thermoelectric systems, the extension of analyses to include other sectors impacted by water scarcity, the creation of decision-support tools for policymakers, utilities, and investors, the examination of dynamic pricing mechanisms to encourage efficient water usage and sustainable energy generation, the participation of stakeholders in discussions related to water and energy, and the investigation of emerging technologies for real-time monitoring and efficient water management.

## Data availability statement

Research data are not shared.

## CRediT authorship contribution statement

**Qiang Guo:** Formal analysis, Data curation, Conceptualization. **Reza Hasani:** Formal analysis, Data curation, Conceptualization.

## Declaration of competing interest

The authors declare that they have no known competing financial interests or personal relationships that could have appeared to influence the work reported in this paper.
